RETRACTED

# One-pot odourless synthesis of thioesters via in situ generation of thiobenzoic acids using benzoic anhydrides and thiourea

**DOI:** 10.3762/bjoc.11.141

**Published:** 2015-07-28

**Authors:** Mohammad Abbasi, Reza Khalifeh

**Affiliations:** 1 Chemistry Department, Faculty of Sciences, Persian Gulf University, Bushehr 75169, Iran; 2 Department of Chemistry, Shiraz University of Technology, Shiraz, Iran

**Keywords:** benzoic anhydride, Michael addition, nucleophilic displacement, thioester, thiourea

## Abstract

An efficient and odourless procedure for a one-pot synthesis of thioesters by the reaction of benzoic anhydrides, thiourea and various organic halides (primary, allylic, and benzylic) or structurally diverse, electron-deficient alkenes (ketones, esters, and nitriles) in the presence of Et_3_N has been developed. In this method, thiobenzoic acids were in situ generated from the reaction of thiourea with benzoic anhydrides, which were subjected to conjugate addition with electron-deficient alkenes or a nucleophilic displacement reaction with alkyl halides.

## Introduction

Thioesters have many uses in organic synthesis as intermediates, mild acyl transfer agents and thiol sources [1–19]. Thioesters can be synthesized in the laboratory by means of different methods using diverse reagents and substrates [20–26]. The reaction of active carboxylic acid derivatives with thiols [27–41] and the coupling of thiols with carboxylic acids using activating agents [42–45] have been mainly used for the synthesis of thioesters in organic synthesis. Thiol-based reactions have a foul smell, making them unpleasant. Thioesters can also be prepared through the conjugate addition and nucleophilic displacement reactions using thioacid nucleophiles. Nevertheless, the reactions of thioacids have not been widely studied because they are not sufficiently available. On the other hand, the usual methods for preparing thioacids involve the action of toxic and unpleasant smelling, gaseous hydrogen sulfide on carboxylic acid derivatives [46–47]. Also, thioacids as thiols have a strong and repulsive smell. The in situ generation of thioacids using odourless, easy to handle and inoffensive substrates is an appropriate solution to these problems. In this regard, the synthesis of *S*-functionalized thioesters using thioaroylate ions in situ generated from acyloxyphosphonium salts and tetrathiomolybdate has been reported [48–50].

## Results and Discussion

The preparation of alkane thiols using thiourea and alkyl halides is a well-known reaction in organic synthesis. In addition, two methods for the synthesis of thioacids from acyl chlorides using *N*,*N*-dimethylthioformamide [51] or thioacetamide [52] have been reported. As far as we know, a similar reaction using thiourea and carboxylic acid derivatives to prepare thioacids has not yet been introduced. Hence, this work is focused on the development of new reaction sequences for the synthesis of thioacid derivatives via in situ generation of thioacids using thiourea as an inexpensive and easy to handle sulfur surrogate.

RETRACTED

Recently, a one-pot procedure for the preparation of thioesters via the reaction of in situ generated thiols (as suggested by other authors) with benzoyl chlorides was reported (Scheme 1, path a) [53]. In this protocol, an alkyl halide was treated with thiourea and a benzoyl chloride in an aqueous Triton X-100 micelle [53]. Alternatively, the thioester could be synthesized from the reaction of the alkyl halide with the thioacid in situ generated from the reaction of thiourea and benzoyl chlorides (Scheme 1, path b).

**Scheme 1:** One-pot procedure for the preparation of thioesters.

In order to explore this possibility, the alkyl halide was removed from the procedure and butyl acrylate was treated with benzoyl chloride and thiourea (Scheme 2). Thiobenzoic acid or its corresponding thia-Michael adduct were not formed after 24 h. The butyl acrylate was intact and the starting benzoyl chloride was mainly converted to potassium benzoate.

**Scheme 2:** Reaction of benzoyl chloride, thiourea and butyl acrylate.

This result confirms that the thioester product cannot be produced through generation of the thioacid from thiourea and benzoyl chloride.

To establish a protocol for the one-pot synthesis of thioacid derivatives via in situ generation of thioacids, considerable preliminary tests were accomplished using thiourea and carboxylic acid derivatives such as esters, acyl halides and anhydrides under various conditions. First, acetyl and benzoyl chlorides were separately treated with an equivalent amount of thiourea by using various solvents and temperatures. The results of these experiments were not satisfactory and after work-up with basic aqueous solutions, a complex mixture of unidentified products was obtained in all experiments. The similar experiments with ethyl acetate and ethyl benzoate did not lead to the formation of any product and the substrates were intact under all experimental conditions tested. Next, a possible reaction between thiourea and carboxylic anhydrides was investigated. As a model reaction, a mixture of well-powdered benzoic anhydride (1 mmol) and thiourea (1.1 mmol) in Et_3_N (0.5 mL) was stirred at 40 °C. The starting benzoic anhydride was gradually consumed within 0.5 h and a two-phase system containing Et_3_N and a thick brick-red liquid was formed. Next, H_2_O (1 mL) and H_2_O_2_ (1.2 mmol) were added to the reaction mixture and the resulting solution was stirred for 1 h at room temperature. Extractive work-up with EtOAc followed by silica gel column chromatography afforded benzoyl disulfide in 91% yield.

RETRACTED

We then focused our attention on developing a practical method to prepare thia-Michael adducts of thioacids. In this regard, a mixture of benzoic anhydride and thiourea in Et_3_N was stirred at 40 °C for 0.5 h. Then, water and *n*-butyl acrylate were added to the mixture and stirring was continued for another 1 h at room temperature. The best results were obtained using 1.3 equiv of thiourea and 1.2 equiv of benzoic anhydride per 1 equiv of butyl acrylate. The desired thia-Michael product was obtained in 86% yield (based on the starting butyl acrylate) and 72% (based on the starting benzoic anhydride) after extractive work-up with EtOAc followed by silica gel column chromatography.

The optimized reaction conditions were then applied to further reactions using structurally diverse benzoic anhydrides and different electron-deficient alkenes. The results are summarized in Table 1.

**Table 1:** One-pot synthesis of thioesters using benzoic anhydrides, thiourea and electron-deficient alkenes^a^.



Entry	R^1^	EWG	*t* (h)	Product	Isolated yield (%)^b^

1	H	COCH_3_	0.5	**1** [48]	80
2	H	CN	0.5	**2** [20]	88
3	H	CO_2_Et	0.5	**3**	90
4	H	CO_2_*n*-Bu	0.5	**4**	86
5	CH_3_	COCH_3_	5	**5**	80
6	CH_3_	CN	5	**6**	84
7	CH_3_	CO_2_Et	5	**7**	88
8	CH_3_	CO_2_*n*-Bu	5	**8**	90
9	Cl	COCH_3_	2	**9**	83
10	Cl	CN	2	**10**	85
11	Cl	CO_2_Et	2	**11**	88
12	Cl	CO_2_*n*-Bu	2	**12**	88
13^c^	CH_3_O	COCH_3_	2	**13**	83
14^c^	CH_3_O	CN	2	**14**	86
15^c^	CH_3_O	CO_2_Et	2	**15**	88
16^c^	CH_3_O	CO_2_*n*-Bu	2	**16**	90

^a^First-step reaction conditions: anhydride (1.2 mmol), thiourea (1.3 mmol), Et_3_N (0.5 mL), 40 °C; Second-step reaction conditions: Micheal acceptor (1 mmol), H_2_O (1 mL), rt. ^b^The yields were calculated based on Michael acceptors as limiting reagents. To achieve yields based on the starting anhydrides or thiourea, they should be divided by 1.2 and 1.3, respectively. ^c^The first step reaction was conducted at 80 °C.

It can be seen that benzoic anhydrides have readily produced the corresponding thioesters through the in situ generation of thioacids. The reaction of aliphatic anhydrides such as acetic, phenylacetic and hexanoic anhydrides with thiourea under the reaction conditions did not lead to the desired thioacids after 24 h. In another project, the optimized reaction conditions were applied to further reactions using structurally diverse benzoic anhydrides and different alkyl halides. The results are shown in Table 2.

RETRACTED

**Table 2:** One-pot synthesis of thioesters using benzoic anhydrides, thiourea and alkyl halides^a^.



Entry	R^1^	R^2^X	*t* (h)	Product	Isolated yield (%)^b^

1	H	*n*-C_10_H_21_I	0.5	**17** [53]	85
2	H		0.5	**18**	90
3	H		0.5	**19** [54]	81
4	H	CH_3_I	0.5	**20**	92
5	H	*n*-C_8_H_17_Br	0.5	**21** [53]	87
6	H		0.5	**22** [55]	90
7	CH_3_		5	**23** [56]	91
8	CH_3_		5	**24**	80
9	CH_3_	*n*-C_8_H_17_Br	5	**25**	84
10	CH_3_	CH_3_I	5	**26** [20]	90
11	CH_3_		5	**27**	90
12	Cl	*n*-C_10_H_21_I	2	**28** [57]	86
13	Cl	CH_3_I	2	**29** [20]	91
14	Cl		2	**30**	87
15	Cl		2	**31**	84
16^c^	CH_3_O		2	**32**	88
17^c^	CH_3_O		2	**33**	81
18^c^	CH_3_O		2	**34**	87
19^c^	CH_3_O	*n*-C_8_H_17_Br	2	**35** [58]	88
20^c^	CH_3_O	CH_3_I	2	**36**	91

^a^First-step reaction conditions: anhydride (1.2 mmol), thiourea (1.3 mmol), Et_3_N (0.5 mL), 40 °C; Second-step reaction conditions: R^2^X (1 mmol), H_2_O (1 mL), rt. ^b^The yields have been calculated based on alkyl halides as limiting reagents. To achieve yields based on the starting anhydrides or thiourea, they should be divided by 1.2 and 1.3, respectively. ^c^The first step reaction was conducted at 80 °C.

As evident from the results presented in Table 2, by this method, primary, benzylic, allylic and propargylic halides have been easily converted to the related thioesters within appropriate reaction times in good to excellent yields (Table 2, entries 1–20).

A general pathway for the reaction has been proposed as presented in Scheme 3. Similar to reactions of acyl chlorides with *N*,*N*-dimethylthioformamide [51] or thioacetamide [52], a benzoic anhydride undergoes a nucleophilic acyl substitution reaction with thiourea to produce the corresponding *S*-benzoylisothiouronium salt as an intermediate. After addition of H_2_O to the reaction mixture, the salt is hydrolyzed by the hydroxide anion to generate the thiobenzoate anion. Finally, the thiobenzoate reacts with a Michael acceptor or an alkyl halide to give the thioester product.

**Scheme 3:** A proposed reaction pathway.

## Conclusion

In conclusion, an efficient, versatile, and odourless protocol for a one-pot preparation of thioesters from non-thiolic precursors under mild conditions has been developed. In this protocol, a mixture of a benzoic anhydride, thiourea and an alkyl halide (primary, allylic or benzylic), or a conjugated olefin (ketones, esters, nitriles), Et_3_N and H_2_O produced the related thioesters in good to excellent yields.

## Experimental

### *S*-3-Oxobutyl benzothioate (**1**)

Colorless oil; ^1^H NMR (250 MHz, CDCl_3_) δ 7.95–7.91 (m, 2H), 7.58–7.52 (m, 1H), 7.45–7.39 (m, 2H), 3.24 (t, *J* = 6.7 Hz, 2H), 2.86 (t, *J* = 6.7 Hz, 2H), 2.16 (s, 3H); ^13^C NMR (62.5 MHz, CDCl_3_) δ 206.5, 191.9, 136.8, 133.5, 128.6, 127.2, 43.4, 29.9, 22.7; IR (neat) *ν* (cm^−1^): 1717 (C=O ketone), 1655 (C=O thioester); anal. calcd for (C_11_H_12_O_2_S): C, 63.43; H, 5.81; S, 15.40; found: C, 63.51; H, 5.77; S, 15.42.

RETRACTED

### Butyl 3-(benzoylthio)propanoate (**4**)

Colorless oil; ^1^H NMR (250 MHz, CDCl_3_) δ 7.95–7.91 (m, 2H), 7.54–7.51 (m, 1H), 7.44–7.38 (m, 2H), 4.09 (t, *J* = 6.6 Hz, 2H), 3.30 (t, *J* = 7.0 Hz, 2H), 2.71 (t, *J* = 7.0 Hz, 2H), 1.65–1.54 (m, 2H), 1.43–1.31 (m, 2H), 0.90 (t, *J* = 7.3 Hz, 3H); ^13^C NMR (62.5 MHz, CDCl_3_) δ 191.5, 171.8, 136.8, 133.5, 128.6, 127.2, 64.7, 34.5, 30.6, 24.1, 19.1, 13.7; IR (neat) *ν* (cm^−1^): 1732 (C=O ester), 1666 (C=O thioester); anal. calcd for (C_14_H_18_O_3_S): C, 63.13; H, 6.81; S, 12.04; found: C, 63.19; H, 6.85; S, 11.98.

### *S*-Decyl benzothioate (**17**)

^1^H NMR (250 MHz, CDCl_3_) δ 7.91–7.86 (m, 2H), 7.51–7.33 (m, 3H), 2.99 (t, *J* = 7.3 Hz, 2H), 1.65–1.54 (m, 2H), 1.38–1.19 (m, 14H), 0.83–0.78 (m, 3H); ^13^C NMR (62.5 MHz, CDCl_3_) δ 192.0, 137.3, 133.1, 128.9, 127.4, 31.9, 29.6, 29.6, 29.5, 29.3, 29.2, 29.0, 29.0, 22.7, 14.1; IR (neat) *ν* (cm^−1^): 1666 (C=O thioester); anal. calcd for (C_17_H_26_OS): C, 73.33; H, 9.41; S, 11.52; found: C, 73.31; H, 9.48; S, 11.46.

### *S*-Prop-2-yn-1-yl benzothioate (**19**)

^1^H NMR (250 MHz, CDCl_3_) δ 7.88–7.84 (m, 2H), 7.53–7.46 (m, 1H), 7.40–7.33 (m, 2H), 3.75 (d, *J* = 2.7 Hz, 2H), 2.15 (t, *J* = 2.7 Hz, 1H); ^13^C NMR (62.5 MHz, CDCl_3_) δ 190.1, 136.2, 133.8, 128.8, 127.3, 78.9, 71.1, 17.5; IR (neat) *ν* (cm^−1^): 3294, 2125, 1670; anal. calcd for (C_10_H_8_OS): C, 68.15; H, 4.58; S, 18.19; found: C, 68.20; H, 4.55; S, 18.26.

### *S*-(2-Methylallyl) 4-methylbenzothioate (**27**)

^1^H NMR (250 MHz, CDCl_3_) δ 7.79 (d, *J* = 8.1 Hz, 2H), 7.14 (d, *J* = 8.1 Hz, 2H), 4.95 (s, 1H), 4.80–4.79 (m, 1H), 3.62 (s, 2H), 2.31 (s, 3H), 1.73 (s, 3H); ^13^C NMR (62.5 MHz, CDCl_3_) δ 191.0, 144.2, 140.9, 134.4, 129.3, 127.3, 114.2, 35.7, 21.7, 21.3; IR (neat) *ν* (cm^−1^): 1659; anal. calcd for (C_12_H_14_OS): C, 69.86; H, 6.84; S, 15.54; found: C, 69.80; H, 6.88; S, 15.61.

## Supporting Information

File 1 Analytical data.

File 2 NMR spectra.
